RETRACTED

# Capsaicin inhibits the migration and invasion via the AMPK/NF-κB signaling pathway in esophagus sequamous cell carcinoma by decreasing matrix metalloproteinase-9 expression

**DOI:** 10.1042/BSR20190819

**Published:** 2019-08-05

**Authors:** Yong Guo, Ning Liu, Kun Liu, Min Gao

**Affiliations:** 1 Office of Drug Purchase, Affiliated Hospital of Jining Medical University, Jining 272000, Shandong, China; 2 Information Technology Centre, Jining Medical University, Jining 272000, Shandong, China; 3 Clinical College, Jining Medical University, Jining 272000, Shandong, China; 4 Clinical Laboratory, Jining No.1 People’s Hospital, Jining 272100, Shandong, China; 5 Jining Medical University, Jining 272011, Shandong, China

**Keywords:** AMPK, Capsaicin, cell invasion, cell migration, ESCC

## Abstract

Antitumor activity of Capsaicin has been studied in various tumor types, but its potency in esophageal squamous cell carcinoma (ESCC) remains to be elucidated. Here, we explored the molecular mechanism of the capsaicin-induced antitumor effects on ESCC Eca109 cells. Eca109 cells were treated with capsaicin *in vitro*, the migration and invasion capacities were significantly decreased by scratch assay and transwell invasion assay. Meanwhile, matrix metalloproteinase (MMP)-9 (MMP-9) expression levels were also obviously down-regulated by Western blot. However, phosphorylated AMPK levels were significantly up-regulated, and this effect was eliminated by the AMPK inhibitor Compound C treatment. In addition, capsaicin can enhance sirtuin1 (SIRT1) expression, which could activate nuclear factor-κB (NF-κB) through deacetylation, and activate AMPK inducing the phosphorylation of IκBα and nuclear localization of NF-κB p65. Overall, these results revealed that Capsaicin can inhibit the migration and invasion of ESCC cells via the AMPK/NF-κB signaling pathway.

## Introduction

Esophageal cancer is one of the most common cancers in the world with high morbidity and mortality [1]. Esophageal cancer is mainly divided into esophageal squamous cell carcinoma (ESCC) and esophageal adenocarcinoma. Although many diagnostic and therapeutic methods have been developed in recent years, whereas a 5-year overall survival rate of ESCC is still less than 14%. Therefore, the development of new therapeutic methods and natural antineoplastic drugs has become an urgent problem in esophageal cancer therapy.

According to previous literature, we know that some of the natural phytochemicals contained in fruits and vegetables have significant inhibitory effects on many cancers at the cellular and molecular levels [2]. Capsaicin (Figure 1A) is one of the phytochemicals present in natural plant peppers and is widely used as a food additive in daily life. Previous studies demonstrated that capsaicin is involved in several physiological and pharmacological effects and anti-proliferative effects on a variety of human cancer cell lines [3–7]. Meanwhile, several studies demonstrate that capsaicin can regulate the survival, inflammation and growth of cancer cells by interfering with the transcriptional activation of nuclear factor-κB (NF-κB) and activator protein-1 (AP-1) [8,9]. However, the mechanism of capsaicin inhibiting the migration and invasion of cancer cells remains unclear.

RETRACTED

**Figure 1:** Capsaicin inhibits proliferation, migration and invasion of Eca109 cells (**A**) This picture represents the chemical structure of capsaicin. (**B**) The viability of Eca109 cells treated with capsaicin (0, 25, 50, 100 μM) for 24 h. (**C,E**) Cell migration was analyzed by a wound healing assay. (**D,F**) Cell invasion was analyzed by transwell assay. *P<0.05 and **P<0.01.

The most difficult reason for patients’ treatment is the invasion and metastasis of tumor cells. Among them, the metastasis mainly involves cancer cells from the primary tumor to the surrounding tissues. In the process of invading the surrounding tissues involves the adhesion of tumor cells, release of extracellular matrix (ECM) degrading enzymes and movement of cancer cells. Interactions between ECM and cells movement exert a direct effect on the whole metastasis process [10]. The matrix metalloproteinase (MMP) family involves the degradation of ECM. Among them, MMP-2 and MMP-9 of MMP family degrade collagen IV during cancer invasion and metastasis. Meanwhile, we found that MMP2 and MMP9 are also expressed in several types of tumor cells [11].

MMP-2 is constitutively expressed in stromal cells, whereas the expression of MMP-9 is induced in both stromal and cancer cells [12,13]. MMP-9 can regulate AP-1, NF-κB and Sp-1 through transcription factors [14]. Cytokines and PMA regulate the activation of transcription factors such as AP-1 and NF-κB to enhance MMP-9 expression [15]. AMPK inhibits NF-κB pathway in mouse embryonic fibroblasts to inhibit MMP-9 expression [16]. Increasing AMPK activation can enhance the activity of sirtuin1 (SIRT1) by increasing cellular NAD^+^ levels [17]. At the same time, deacetylation of the NF-κB p65 by SIRT1 inhibits NF-κB signaling [18,19], indicating that SIRT1 can decrease the expression of MMP-9 by deacetylation of NF-κB [20,21].

In short, our study investigated whether capsaicin can inhibit the migration and metastasis in ESCC cells via the AMPK/NF-κB signaling pathway.

## Materials and methods

### Cell line and reagents

Human ESCC Eca109 cell lines were purchased from the Type Culture Collection of the Chinese Academy of Sciences (Shanghai, China), cultured in RPMI-1640 medium supplemented with 10% fetal bovine serum (HyClone, Utah, U.S.A.), 100 U/ml penicillin and 100 μg/ml streptomycin (Invitrogen), and incubated at 37°C and 5% CO_2_. Capsaicin was purchased from Sigma (St. Louis, MO, U.S.A.). Anti-MMP-2, anti-MMP-9, anti-AMPK, anti-p-AMPK, anti-SIRT1, anti-p65, anti-lamin A, anti-IκBa, anti-p-IκBa, α-tubulin and anti-β-actin were obtained from Santa Cruz Biotechnology (Santa Cruz, CA, U.S.A.).

RETRACTED

### Cell proliferation assay

Eca109 cells (2 × 10^3^ cells/well) were incubated in 96-well plates, and cells were treated with various concentrations of capsaicin (0, 25, 50, 100 μM). After incubation for 24 h, 10 μl cell counting kit-8 (CCK-8) solution (Promega, Fitchburg, WI, U.S.A.) was added to each well and the mixture was incubated at 37°C, 5% CO_2_ incubator for 1 h, then the absorbance was measured by microplate reader at 450 nm wavelength.

### Wound healing assay

Cells (5 × 10^5^/well) were cultured in six-well plates until monolayers were formed. A scratch was created using 10 μl pipette tip in each well. Then, capsaicin added to each well for 24 h. Pictures were collected at 0 and 24 h in the presence and absence of capsaicin to observe cell migration closure using inverted microscope (Thermo Fisher Scientific, Inc).

### Cell invasion assay

We assayed the invasion ability of cells using 6.5 mm diameter Transwell chambers with 8-μm membranes (Corning, U.S.A.). Cells (5 × 10^4^) were incubated into upper chamber, and the bottom wells were coated with 1 mg/ml Matrigel for the invasion assays, whereas the RPMI-1640 medium consisting of 10% FBS was supplemented to the lower chamber. After incubation for 24 h, the cells remaining on the upper membrane were discarded with cotton swab. The membrane were fixed in 4% polyformaldehyde and stained with 0.1% Crystal Violet for 15 min at 4°C. Finally, invaded cells number were counted using photographic images.

### Quantitative reverse-transcription polymerase chain reaction

Total RNAs were obtained from cells using TRIzol reagent (Solarbio, Beijing, China). Two micrograms of total RNA was performed to synthesize cDNA using PrimeScript RT Reagent Kit (Takara, Dalian, China). Then, PCR amplication was performed with GFX96 real-time PCR system (Thermo Fisher Scientific, U.S.A.). Bar diagram presented the relative expression normalized to GAPDH. Results were calculated using the 2^−ΔΔ*C*^_t_ method.

### Gelatin zymography

Conditioned medium and cell lysates were electrophoresed in a polyacrylamide gel supplemented with 1 mg/ml gelatin. Subsequently, the gel was washed with 2.5% Triton X-100 for 2 h, and transferred to a buffer at 37°C overnight. Finally, the gel was stained with 0.2% Coomassie Blue staining solution. Proteolysis was analyzed as a dark zone in the gray-white area.

RETRACTED

### Immunoblot analyses and immunoprecipitation

For immunoblotting, nuclear protein (500 μg) and antibody–conjugated resin were incubated overnight at 4°C. Then, the unbound protein was removed by centrifugation, and the resin was washed with the immunoprecipitation (IP) lysis, and antigen was eluted with elution buffer. Protein was isolated by SDS/PAGE, and transferred to PVDF membrane. Finally, bands were measured using chemiluminescence ECL detection system. Band intensity was analyzed using the ImageJ software.

### Chromatin IP

Cell extract was pre-cleared by incubation with protein A-agarose/salmon sperm DNA at 4°C overnight. Then, incubated with NF-κB p65 antibody. After precipitation, the antibody–chromatin complex was transferred to spin column, and washed three times with different buffers, such as low-salt, high-salt, LiCl, high-salt LiCl immune complex wash buffer and Tris/EDTA buffer. Subsequently, protein–DNA complexes were eluted with elution buffer so that DNA was detached from the complex. DNA was analyzed by PCR using promoter-specific primer pairs for the NF-κB binding site of the MMP-9 promoter (forward: 5′-GCCATGTCT GCTGTTTTCTAGAGG-3′, and reverse: 5′-CACACTCCAGGCTCTGT CCTCTTT-3′).

### Statistical analysis

All the statistical analysis was performed using the Student’s *t* test by SPSS 22.0 software (SPSS Inc., Chicago, IL, U.S.A.). All the quantitative data are expressed as means ± standard deviation. A probability value of *P*<0.05 was considered to indicate statistically significant difference.

## Results

### Inhibition of Capsaicin on the proliferation of ESCC cells

CCK-8 assay was determined at 24 h after capsaicin treatment at different concentrations (0, 25, 50 and 100 μM). The results were shown in Figure 1B, capsaicin inhibited the proliferation of Eca109 cells (*P*<0.05). Therefore, safe concentrations of capsaicin (50 μM) for 24 h was selected.

### Capsaicin restricts the migration and invasion of ESCC cells

Wound healing and Transwell invasion experiment were carried out. Number of migration and invasion were analyzed after capsaicin treatment (50 μM) for 24 h. The results demonstrated that the migration (Figure 1C,E; *P*<0.05) and invasion (Figure 1D,F; *P*<0.05) ability of Eca109 cells treated with capsaicin were significantly suppressed, suggesting that capsaicin can inhibit the growth, migration and invasion ability of Eca109 cells.

### Capsaicin decreases the expression of MMP-9

Previous research has confirmed that MMP expression plays an important role in local proteolysis of the ECM and cell migration [22]. Therefore, our results indicated that the protein expression of MMP-9 and MMP-2 were remarkerly reduced compared with control groups in the capsaicin-treated cells (Figure 2A–C,G; *P*<0.05). while, this result is consistent with that induced by PMA at 48 h (Figure 2D–F; *P*<0.05). Our results also found that capsaicin can significantly down-regulate MMP-2 and MMP-9 mRNA expression by real-time quantitative PCR (RT-qPCR) (Figure 2H–J; *P*<0.05). In short, our results demonstrated that capsaicin can inhibit MMP-2 and MMP-9 expression.

RETRACTED

**Figure 2:** Capsaicin inhibits MMPs production in Eca109 cells (**A**–**C**) MMP-9 and MMP-2 expression in Eca109 cells treated with capsaicin were detected by immunoblot assay. (**D**–**F**) MMP-9 and MMP-2 in Eca109 cells pretreated with PMA (20 nM) were detected by immunoblot assay. (**G**) MMP-9 and MMP-2 in Eca109 cells culture supernatants were analyzed by gelatin zymography. (**H**–**J**) MMP-9 and MMP-2 in cell extracts were analyzed by RT-qPCR. **P<0.01.

### Capsaicin activates AMPK to regulate MMP-9 expression

Previous study demonstrated that MMP-9 expression was related to AMPK activation [16]. Our study was to explore whether capsaicin can activate AMPK in the Eca109 cells, as illustrated in Figure 3. Capsaicin (50 μM) can significantly enhance the protein level of p-AMPK (Figure 3A; *P*<0.05). However, we did not know whether increasing p-AMPK expression affected the expression of MMPs. Then, with capsaicin followed by compound C treated the cells. Our results demonstrated that Compound C can reverse the MMP-9 protein expression, as shown in immunoblotting (Figure 3B; *P*<0.05) and gelatin zymography (Figure 3C; *P*<0.05), suggesting that MMP-9 expression down-regulation by capsaicin is mediated via AMPK activation.

**Figure 3:** Capsaicin inhibits MMP-9 expression via activating AMPK signaling pathway in Eca109 cells (**A**) p-AMPK in capsaicin-treated cells was analyzed by immunoblot assay. (**B,C**) Immunoblot analysis (B) and gelatin zymography (C) of MMP-9 in cells treated with capsaicin and with an AMPK inhibitor (compound C). *P<0.05 and **P<0.01.

### SIRT1 is responsible for the inhibition of capsaicin by activating AMPK

SIRT1 as a protein deacetylase is considered to decrease MMP-9 expression by switching off its expression [20], as shown in Figure 4. Capsaicin treatment significantly increased the protein expression of SIRT1 in the Eca109 cells (Figure 4A; *P*<0.05), whereas Sirtinol, a SIRT1 inhibitor, reversed the MMP-9 expression and activity (Figure 4B,C; *P*<0.05). Subsequently, we also found that AMPK and SIRT1 inhibitor abolished the capsaicin-induced change (Figure 5A–D; *P*<0.05), suggesting that AMPK-mediated deacetylation of SIRT1 is associated with the inhibition of MMP-9 expression by capsaicin.

RETRACTED

**Figure 4:** Capsaicin increases SIRT1 levels via activating AMPK signaling pathway in Eca109 cells (**A**) SIRT1 in the capsaicin-treated cells was analyzed by immunoblot assay. (**B**) MMP-9 protein levels. (**C**) Gelatin zymography of MMP-9. Cells were treated with Sirtinol (1 μM) or Compound C (1 μM) followed by 50 μM capsaicin for 24 h. *P<0.05 and **P<0.01.

**Figure 5:** AMPK-SIRT1 signaling mediates the inhibitory effect of capsaicin on the migration and invasion of Eca109 cells (**A,C**) Capsaicin-treated Eca109 cells also exposed to compound C or sirtinol were analyzed by wound healing assay. (**B,D**) Capsaicin-treated Eca109 cells were analyzed by transwell assay. Cells were treated with Sirtinol (1 μM) or Compound C (1 μM) followed by 50 μM capsaicin for 24 h. **P<0.01.

### NF-κB is involved in the capsaicin-induced MMP-9 expression down-regulation

According to the previous literature and the above experiments, we speculated whether capsaicin-induced activation of AMPK influences the nuclear translocation of the NF-κB subunit p65. Our results showed that NF-κB p65 protein levels were significantly decreased in the nucleus but increased in the cytoplasm (Figure 6A; *P*<0.05) without capsaicin treatment. However, this effect was abolished by the AMPK inhibitor treatment. Meanwhile, our study also found that capsaicin obviously decreased the level of p-IκBa (Figure 6B; *P*<0.05), and this effect was abolished by AMPK inhibitor treatment, suggesting that p-IκBa expression levels were regulated through the capsaicin-induced AMPK signaling pathway. To determine whether capsaicin activated the deacetylation of p65 by SIRT1. We observed that capsaicin significantly promoted specific SIRT1 protein binding to p65, and to reduce levels of acetyl-p65 protein (Figure 6C; *P*<0.05). Our results found that capsaicin’s effect was blocked by compound C or Sirtinol treatment, suggesting that capsaicin-induced AMPK activiation affects the deacetylation and nuclear translocation of the NF-κB p65, which ultimately leads to inhibition of MMP-9 expression.

**Figure 6:** Capsaicin inhibits the activity of the NF-κB subunit p65 via the SIRT1- or IBa-mediated signaling pathway (**A**) NF-κB p65 expression in capsaicin-treated cells was analyzed by immunoblot assay. Cytosolic and nuclear fractions were subjected to immunoblotting using anti-NF-κB p65 antibody or anti-lamin A antibody (as a nuclear control). (**B**) p-IκBa expression in capsaicin-treated cells was analyzed by immunoblot assay. (**C**) SIRT1 and acetyl-NF-κB p65 expression after IP with NF-κB p65 was analyzed by Immunoblot assay. Cells were treated with Sirtinol (1 μM) or Compound C (1 μM) followed by 50 μM capsaicin for 24 h. *P<0.05 and **P<0.01.

RETRACTED

### Capsaicin decreases the recruitment of NF-κB p65 to MMP-9 promoter region

As shown in Figure 7, Capsaicin decreased the recruitment of NF-κB p65 to the MMP-9 promoter region (Figure 7A–F; *P*<0.05). Then, we also observed that capsaicin can decrease the binding of p300 acetyltransferase, which regulates the acetylation of NF-κB p65 in MMP-9 transcription [23]. However, the binding of SIRT1 deacetylase was significantly decreased after capsaicin treatment cells, which was blocked by compound C or Sirtinol treatment, indicating that capsaicin decreased the recruitment of NF-κB p65 to MMP-9 promoter region through AMPK-associated deacetylation of SIRT1. Therefore, we demonstrated that the deacetylation of p65 by SIRT1 and the nuclear translocation of p65 induced by IκBa phosphorylation are responsible for the MMP-9 gene expression promoted by p65 after capsaicin treatment cells.

**Figure 7:** Capsaicin reduces the recruitment of the transcription factor NF-κB p65 to the MMP-9 promoter region (**A**) Immunoblot analysis of IgG, Input, Ac-lysine, p300, NF-κB p65 and SIRT1. Chromatin IP (ChIP) assays were conducted using anti-IgG (**B**), ac-lysine (**C**), p300 (**D**), NF-κB p65 (**E**), SIRT1 (**F**) antibodies. The input (as a negative control) represents PCR products from chromatin pallets prior to immunoprecipitation. **P<0.01.

## Discussion

Capsaicin is a naturally occurring plant phytochemical present in chili peppers. Whether it acts as a carcinogen, co-carcinogen or anti-carcinogen is controversial [24,25]. Nevertheless, accumulating findings indicate that capsaicin has anti-cancer properties in various cancer cell lines. The purpose of the present study was to explore the mechanism of capsaicin-induced cell death in human Eca109 cancer cells. Here, we report that capsaicin-treated Eca109 cells inhibit their viability, migration and invasion, and down-regulate MMP-9 expression via AMPK-NF-κB signaling pathway.

Due to lymph node metastases, deep tumor infiltration and early diagnosis difficulty, most patients with esophageal cancer have a relatively low survival rate [26,27]. Conventional chemotherapy and radiation are ineffective in prolonging the long-term survival of patients with these cancers unless the tumors are removed by complete surgical resection. Therefore, it is crucial to find new treatments and strategies. Recently, there have been extensive studies on capsaicin in tumor cells. Studies have shown that capsaicin can inhibit the migration of various tumor cells [28]. In this study, we explored that capsaicin can inhibit the migration and invasion of esophageal cancer Eca109 cells, and studied its mechanism.

RETRACTED

Previous studies have shown that MMPs are involved in the process of cancer cell migration and metastasis [13,29]. In this study, MMP-9 mRNA and protein levels were significantly decreased in Eca109 cells after capsaicin treatment. Therefore, we hypothesized that the regulation of MMP-9 transcription contributes to the inhibition of capsaicin on cell migration and invasion, and regulated by binding transcription factors NF-κB and AP-1 to MMP-9 promoter region [14]. Capsaicin interference transcription factors such as NF-κB and AP-1 induced activation, thereby reducing the survival of various cell types, inflammation and growth [9]. Meanwhile, our results shown that capsaicin suppressed translocation of NF-κB p65 to the nucleus and its binding to the MMP-9 promoter sequences. In short, capsaicin down-regulates MMP-9 expression by regulating NF-κB in the Eca109 cells. Nuclear translocation of NF-κB is activated by phosphorylation and dissociation of IκBa from the NF-κB complex in the cytoplasm. Our results indicated that capsaicin inhibited p-IκBa expression.

In another way, activation of NF-κB can also be achieved through AMPK, mainly by increasing the concentration of intracellular NAD^+^, thereby activating the NAD^+^-dependent deacetylase SIRT1, which ultimately leads to the deacetylation of the SIRT1 target NF-κB [18]. In our study, capsaicin can regulate the deacetylation of p65 in Eca109 cells. However, SIRT1 inhibitor treatment reversed the effect of capsaicin. Studies have shown that acetylated p65 by p300 causes a change in the transcriptional activity of its MMP-9 expression [30]. Thus, SIRT1-mediated deacetylation and IκBa-mediated nuclear translocation may be associated with capsaicin effect on MMP-9 expression through NF-κB signaling. Two pathways are known to independently regulate the transcription factor NF-κB, they are co-regulated by AMPK, suggesting that the AMPK-mediated signaling pathway was involved in capsaicin action. Meanwhile, TRPV1 activation significantly up-regulated the phosphorylation of AMPK by capsaicin treatment [31]. In our study, capsaicin increased AMPK activation, levels of NAD^+^ and SIRT1 by phosphorylation, while Compound C showed the opposite effect. At the same time, Compound C reversed the anti-migration and anti-invasion effects of capsaicin. These results provide evidence that capsaicin affects AMPK activation upstream of NF-κB signal transduction. In addition, a telomeric protein Rap1 (repressor/activator protein) acts as a regulator of the NF-κB signaling through promoting IKK-mediated p65 phosphorylation, leading to the activation of NF-κB target genes expression and regulating the inflammatory response [32–34]. Depletion of endogenous DDX20 (belongs to the family of DEXD/H-box proteins) in invasive cancer cells led to decreased expression of matrix metallopeptidase 9 (MMP9) and impeded cell migration and invasion. Mechanistic studies showed that DDX20 is a critical cofactor for TAK1-mediated activation of IKK2, the key NF-B-activating kinase in its activation loop [35]. Increasing reports have focused on a family of proteins known as DEAD/H-box helicases involved in RNA metabolism, regulation of long and short noncoding RNAs, and novel roles as ‘editing Helicases’ and their association with cancers [36]. In addition, DEAD/H-box helicases may act as a potential pharmacological drug targets in cancers. These findings will provide new ideas for our future research.

RETRACTED

In conclusion, our results demonstrated that capsaicin retrains the invasion and migration of Eca109 cells by inhibiting NF-κB p65 via the AMPK-SIRT1 and the AMPK-IκBa signaling pathways, which cause MMP-9 expression inhibition.

## Abbreviations

AP-1: activator protein-1
CCK-8: cell counting kit-8
ECM: extracellular matrix
ESCC: esophagus sequamous cell carcinoma
MMP: matrix metalloproteinase
NF-κB: nuclear factor-κB
SIRT1: sirtuin 1
